# Clinical Observation of Levothyroxine Sodium Combined with Selenium in the Treatment of Patients with Chronic Lymphocytic Thyroiditis and Hypothyroidism and the Effects on Thyroid Function, Mood, and Inflammatory Factors

**DOI:** 10.1155/2021/5471281

**Published:** 2021-10-27

**Authors:** Chunping Sun, Min Zhu, Li Li, Hua Fan, Fang Lv, Defa Zhu

**Affiliations:** ^1^Department of Endocrinology, The First Affiliated Hospital of Anhui Medical University, Anhui Gerietric Institute, Hefei, Anhui 230022, China; ^2^Department of Endocrinology, The Third Affiliated Hospital of Anhui Medical University, Hefei, Anhui 230022, China

## Abstract

The purpose of this study was to investigate the therapeutic effects of levothyroxine sodium combined with selenium treatment and single levothyroxine sodium treatment on patients with chronic lymphocytic thyroiditis and hypothyroidism and to analyze the effects of different treatment regimens on patients' thyroid function, mood, and inflammatory factors, with the aim of providing a reference for clinical treatment. The subjects of the current study were 138 chronic lymphocytic thyroiditis (CLT) patients with hypothyroidism admitted to our hospital from May 2016 to September 2019 and were randomly divided into a control group taking levothyroxine sodium (LT4) treatment and a combined group of LT4 combined with selenium treatment, with 69 cases each. Patients in both groups were evaluated for efficacy after 3 months of treatment, and their thyroid function was observed by total triiodothyronine (TT3), total thyroxine (TT4), thyroid stimulating hormone (TSH), thyroid peroxidase antibody (TPOAb), and thyroid globulin antibody (TGAb), and their mood changes were observed by Self-Rating Anxiety Scale (SAS) and Self-Rating Depression Scale (SDS) scores. The levels of inflammatory factors such as interleukin-2 (IL-2), interleukin-10 (IL-10), and tumor necrosis factor-*α* (TNF-*α*) were measured, and the occurrence of adverse drug reactions during the treatment period was observed and recorded in all patients. The results showed that the total effective rate of the combined group was significantly higher than that of the control group. The levels of TT3, TT4, TSH, TgAb, and TPOAb, SAS and SDS scores, and levels of inflammatory factors such as IL-2, IL-10, and TNF-*α* were significantly improved in both groups after treatment. Compared with the control group, TGAb, TPOAb, IL-2, TNF-*α* levels, and SAS and SDS scores decreased more and IL-10 levels increased more in the combined group, while the differences of other indexes were not statistically significant. This suggests that LT4 has certain efficacy in treating CLT with hypothyroidism, and the combined selenium treatment can improve the therapeutic effect of LT4 and can play a greater role in improving patients' mood and immune and inflammatory responses.

## 1. Introduction

Chronic lymphocytic thyroiditis (CLT), also known as Hashimoto's thyroiditis, is an autoimmune disease characterized by diffuse goiter infiltrated by lymphocytes and is the leading cause of hypothyroidism in iodine-sufficient regions of the world [1, 2]. The disease develops slowly and its clinical manifestations are not specific. In the early stage, the thyroid function of patients is mostly normal or hyperthyroid, but with the further development of the disease, the thyroid tissue is heavily damaged and its ability to synthesize and release thyroid hormones is reduced, which can lead to hypothyroidism and cause disorders of lipid metabolism in patients and reduce their quality of life [3]. The pathogenesis of CLT is not fully understood and is thought to be triggered by a combination of genetic, immune, and environmental factors. It has been suggested that systemic immune inflammatory factors are also involved in the development of CLT and that imbalance of the helper type 1 (Th1)/Th2 ratio is closely related to the development of CLT [4, 5].

Thyroid hormone deficiency can lead to emotional and cognitive abnormalities, and patients can present with mild depression and anxiety or significant psychiatric disorders. Severe cases can eventually enter a state of psychosis if they are left untreated or mishandled [6]. At present, the common clinical treatment for CLT patients with hypothyroidism is thyroid hormone alternative therapy, which can alleviate a series of clinical symptoms manifested by hypothyroidism. However, there are still some patients who are unable to effectively control the progression of the disease, resulting in increasingly severe symptoms of hypothyroidism [7, 8]. More studies have shown [9, 10] that selenium deficiency in vivo is closely related to the development of CLT and that selenium plays an important regulatory role in the thyroid antioxidant system and immune disorders. Selenium, as one of the essential trace elements, is present in almost all immune cells, has immunomodulatory effects, and is abundant in thyroid tissue, and selenium deficiency in the body affects normal thyroid secretion [11]. Studies have confirmed [12] that plasma selenium levels are significantly lower in patients with CLT than in the normal population and that clinical efficacy has been achieved with selenium in the treatment of thyroid disorders. It has also been shown [13] that low selenium intake is associated with increased risk of depressed mood and major depression in women and that moderate dietary selenium intake can improve mood in the general population.

We therefore used levothyroxine sodium (LT4) combined with selenium and LT4 alone to treat patients with CLT and hypothyroidism, and we observed changes in thyroid function, anxiety and depression, and inflammatory factors in patients of different treatment regimen groups to investigate the effect of selenium supplementation on patients with CLT and hypothyroidism.

## 2. Materials and Methods

### 2.1. Materials

138 CLT patients with hypothyroidism admitted to our hospital from May 2016 to September 2019 were selected, including 44 males and 94 females. Subjects were numbered 1 to 138 according to the time of enrollment, and the patients were divided into 69 cases each in the control group treated with LT4 and the combined group of LT4 combined with selenium treatment according to the random number table method. General data such as age, duration of disease, body mass index (BMI), degree of goiter, history of smoking, and history of alcohol abuse were collected and compared between the two groups. The results showed that there was no statistically significant difference between the general data of the two groups (*P* > 0.05, Table 1), and they were comparable.

### 2.2. Grading of the Degree of Goiter

Mild: the enlarged thyroid gland in the neck cannot be observed by the naked eye, but the thyroid gland can be palpated by palpation. Moderate: the enlarged thyroid gland in the neck can be seen with the naked eye, and the outline of the enlargement can be palpated, but the enlarged thyroid gland does not exceed the posterior border of the sternocleidomastoid muscle. Severe: the thyroid gland is visually and palpably enlarged and extends beyond the posterior border of the sternocleidomastoid muscle.

### 2.3. Diagnostic Criteria for CLT [14]

Diagnostic criteria for CLT were defined as follows: (1) thyroid peroxidase antibody (TPOAb) > 60 U/ml and thyroid globulin antibody (TGA) > 60 U/ml; (2) color Doppler ultrasound showing diffuse thyroid lesions rather than thyroid nodules or other lesions; and (3) thyroid fine needle aspiration and cytology consistent with the pathological manifestations of CLT. The diagnosis was confirmed if (1) + (2) or (2) + (3) was met.

### 2.4. Diagnostic Criteria for Hypothyroidism [15]

Diagnostic criteria for hypothyroidism were defined as follows: (1) decreased metabolic rate and decreased sympathetic excitability are the main clinical manifestations. (2) Laboratory tests reveal elevated serum thyroid-stimulating hormone (TSH) and decreased total thyroxine (TT4) and free thyroxine (FT4); serum total triiodothyronine (TT3) and free triiodothyronine (FT3) are decreased in the late stage.

### 2.5. Inclusion Criteria

Patients were included if they (1) met the above diagnostic criteria; (2) aged from 20 to 64 years; (3) did not combine with serious cardiovascular, cerebrovascular, hepatic and renal system, and hematopoietic system diseases and psychiatric disorders; (4) did not receive thyroid hormone and immunomodulatory preparations and selenium preparations in the 1 month prior to enrollment; (5) had no comorbid autoimmune diseases; and (6) were informed and agreed to participate in the study.

### 2.6. Exclusion Criteria

Exclusion criteria were as follows: (1) those with obvious gastrointestinal disorders who were not suitable for oral medication; (2) women who were pregnant, lactating, or planning to become pregnant within six months; (3) those who were allergic or hypersensitive to the medication used in the study; and (4) those with other combined thyroid disorders.

### 2.7. Withdrawal and Exclusion Criteria

Withdrawal and exclusion criteria were as follows: (1) those who did not use the drugs as prescribed, violate the treatment protocol, use other drugs in combination, etc., which affect the clinical efficacy and safety evaluation, were excluded. (2) Those who did not complete the treatment course and observation period specified in the protocol due to adverse reactions, ineffectiveness, loss of patient visits, automatic withdrawal, etc., were considered as dropped cases.

### 2.8. Treatment Method

Control patients received oral treatment with LT4 (Merck KGaA, approval number H20100523, Germany) at an initial starting dose of 25 to 50 *μ*g/d before meals. Thyroid function tests were then performed every 2 weeks, and the dose was adjusted to increase by 25–50 *μ*g according to the results of the tests and the patient's specific condition, with a maintenance dose of 50–100 *μ*g taken once a day before meals for 3 months of continuous treatment. In the combined group, the LT4 treatment was the same as that in the single treatment group, with additional selenium supplementation treatment, selenium yeast tablets (produced by Jilin Yinoke Pharmaceutical Co., Ltd., approval number H10940161) orally, 50 *μ*g/d time, 2 times/d, for 3 months.

### 2.9. Observation Indicators

1. Serum index test: all patients were registered by the same physician with name, age, and duration of thyroid disease, and venous blood was drawn by the same nurse the next morning after 12 h fasting. In each group, 5 ml of venous blood was drawn from the fasting elbow before and after the treatment, and the test was performed by our laboratory for thyroid function such as TT3, TT4, and TSH, autoimmune antibodies such as TPOAb and TgAb, and plasma immunoinflammatory factor interleukin-2 (IL-2), interleukin-10 (IL-10), and tumor necrosis factor-*α* (TNF-*α*) were measured. TT3, TT4, and TSH levels were measured by radioimmunoassay kits. Serum TgAb and TPOAb were determined by electrochemiluminescence immunoassay, and serum IL-2, IL-10, and TNF-*α* were detected by enzyme-linked immunosorbent assay. Normal reference values are in the following ranges: TT3: 0.92–2.79 nmol/l, TT4: 58.10–161.30 nmol/l, TSH: 0.27–4.780 mU/l, TPOAb < 60 U/ml, TgAb < 60 U/ml, IL-2: 1.5∼2 ng/L, IL-10: (38.6 ± 10.6) ng/ml, and TNF-*α* <90 mg/L.
2. Emotional assessment: all scales were assessed before and after treatment by dedicated personnel. The Self-Rating Anxiety Scale (SAS) contains 20 subquestions, each divided into 4 options: no or little time, a small amount of time, a considerable amount of time, and most or all of the time, which the participant checks off on a paper-based scale. Subjects were told to take care to understand each question description and not to make multiple choices or omit choices. Assess the actual feeling of the past week honestly, try to complete each form within 10 minutes, and ask for help from the supervisor if you encounter problems such as problem descriptions that you cannot understand, and the supervisor must not give guidance to the subject. The raw score obtained by the staff was multiplied by 1.25 and the integer part of the result was set as the standard score. The standard score cut-off was 50 points, with mild anxiety at 50 to 59 points, moderate anxiety at 60 to 69 points, and severe anxiety >70 points. The standard score of Self-Rating Depression Scale (SDS) was 53 points, 53 to 62 points for mild depression, 63 to 72 points for moderate depression, and >72 points for severe depression.
3. Occurrence of adverse drug reactions: the occurrence of adverse reactions such as nausea, fever, dizziness, chest tightness, and bloating occurring during the treatment period in the two groups was recorded and compared. The incidence of total adverse reactions = (nausea + fever + dizziness + chest tightness + bloating) cases/total cases × 100%.

### 2.10. Efficacy Evaluation

The clinical efficacy of the patients was evaluated at the end of the treatment and was divided into 3 grades. Markedly effective: clinical symptoms and signs disappeared after treatment, with no goiter, and the indexes of laboratory tests returned to normal. Efficient: clinical symptoms and signs improved significantly, nodules subsided or became softer and smaller, goiter pain was reduced, TGAb or TPOAb turned negative or had a decreasing trend, and thyroid function was basically normal. Invalid: the effective standard was not reached, thyroid nodules or enlargement still existed, TGAb or TPOAb did not change, or the condition deteriorated. Total effective rate = number of (markedly effective + efficient) cases/total cases × 100%.

### 2.11. Statistical Methods

SPSS 20.0 statistical software was used to statistically analyze the data, and Prism 8.0 was used for graphing. The statistical data were expressed as (*n*, %) by chi-square test (*χ*^2^), and nonparametric tests (*z*) were used for grade information. The measurement data were expressed as mean ± standard deviation (mean ± SD), and according to the normality test, *t*-test was used for conformity to normality, and rank sum test was used for nonconformity. *P* < 0.05 indicated a statistical difference.

## 3. Results

### 3.1. Comparison of Clinical Efficacy

After 3 months of treatment, 5 cases were shed in the control group, and 64 cases finally completed the experiment; 4 cases were shed in the combined group, and 65 cases finally completed the experiment. The efficacy of the two groups was evaluated at the end of treatment. In the control group, 38 cases were markedly effective, 15 cases were efficient, and 11 cases were invalid, and the total effective rate of this group was 82.81% (53/64). In the combined group, there were 45 cases with markedly effective, 17 cases with efficient, and 3 cases with invalid evaluation, and the total effective rate of this group was 95.38% (62/65). A comparison of the total effective rate of the two groups showed that the combined group was significantly higher than the control group (*P* > 0.05, Figure 1).

### 3.2. Comparison of Thyroid Function before and after Treatment

The TT3, TT4, TSH, TPOAb, and TGAb levels before treatment were compared between the two groups, and the differences were not statistically significant (*P* > 0.05). After treatment, TT3 and TT4 levels increased and TSH, TPOAb, and TGAb levels decreased in both groups (*P* < 0.05). Compared with the control group, TPOAb and TGAb levels decreased more in the combined group (*P* < 0.05), and the differences in other indexes were not statistically significant (*P* > 0.05) (Figure 2).

### 3.3. Comparison of SAS and SDS Scores before and after Treatment

The differences in SAS and SDS scores between the two groups at pretreatment were not statistically significant (*P* > 0.05) and were in the high range, which suggested that both CLT hypothyroid patients had some emotional problems. After treatment, SAS and SDS decreased in both groups, of which the combined group were significantly lower than the control group (*P* < 0.05) (Figure 3), which suggested that LT4 combined with selenium supplementation could improve patients' mood more effectively.

### 3.4. Comparison of Inflammatory Factor Levels before and after Treatment

The levels of IL-2, IL-10, and TNF-*α* were similar in both groups before treatment, and the differences were not statistically significant (*P* > 0.05). After treatment, the levels of IL-2 and TNF-*α* in the two groups were significantly lower than those before treatment, while the level of IL-10 was significantly higher. Among them, IL-2 and TNF-*α* levels in the combined group were lower than those in the control group, and IL-10 levels were higher than the control group, and the difference was statistically significant (*P* < 0.05) (Figure 4).

### 3.5. Comparison of the Occurrence of Adverse Reactions

The adverse drug reactions that occurred during the treatment were counted in both groups. In the control group, there were 2 cases of nausea, 3 cases of fever, 2 cases of dizziness, 1 case of chest tightness, and 3 cases of bloating, with a total incidence of 17.19% (11/64). In the combined group, there were 1 case of nausea, 2 cases of fever, 1 case of dizziness, 2 cases of chest tightness, and 2 cases of bloating, with a total incidence of 12.31% (8/65). The total incidence of adverse reactions was compared between the two groups, and the difference was not statistically significant (*P* > 0.05, Figure 5).

## 4. Discussion

CLT is an organ-specific autoimmune disease in which the thyroid is the main target organ of immune damage, and pathological examination reveals a massive diffuse infiltration of lymphocytes in the thyroid parenchyma with a predominance of helper T cells (Th). Repeated thyroid follicular epithelial destruction and fibrous tissue hyperplasia eventually result in subclinical hypothyroidism (SCH) [16, 17]. If left untreated, 5% of CLT patients with SCH may convert to clinical hypothyroidism (OVH) each year, aggravating the patient's condition [18]. LT4 is currently used as replacement therapy in CTL patients with hypothyroidism to prevent the progression of SCH to OVH and to prevent SCH and OVH-related complications [19].

The application of exogenous LT4 can supplement the insufficient secretion of thyroid hormones in the patient's organism, but it does not significantly improve antibody titers such as TPOAb, thus leading to a high relapse rate in patients after treatment [20]. The main feature of CLT is the detection of highly potent antithyroid antibodies in the blood, which is an important reason for calling it an autoimmune disease. TPOAb and TGAb are important landmark antibodies in HT, and the detection of both usually marks the body's immune dysfunction [21]. In this study, patients in both groups had significantly high levels of TPOAb and TGAb before treatment, which suggested the prevalence of immune disorders in patients with CLT and hypothyroidism. After treatment, the antibody levels in both groups decreased significantly, with lower levels in the combined group; and the overall effective rate in the combined group was significantly higher than that in the control group. Selenium is an essential trace element and is one of the essential daily dietary nutrients, which has the functions of antioxidant, immune enhancing, antagonistic to toxic substances, maintains the growth and development of several organs of the body, and is essential for maintaining the homeostasis of the endocrine system immune, metabolism, etc. [22]. When there is selenium deficiency, disruption of the body's immune system, weakened antioxidant effect, and insufficient scavenging of free radicals lead to the destruction of thyroid follicular epithelial cells and the release of Tg and TPO into the circulation, which triggers an immune inflammatory response and a significant increase in the body's TPOAb and TGAb levels, thus inducing or aggravating CLT [23, 24]. Therefore, the treatment with selenium supplementation can reduce the level of TPOAb and TGAb and prevent further destruction of thyroid tissue, which can enhance the effect of LT4 replacement therapy. Some studies showed that selenium supplementation therapy could improve the levels of thyroid function-related indexes in CLT hypothyroid patients, while in this study, TT3, TT4, and TSH were improved in the control and combined groups after treatment but the difference between the two groups was not significant, which might be related to the short observation time of the experiment.

Current studies have indicated [25, 26] that Th1/Th2 cytokine immune imbalance plays an important role in the development of CLT and is mainly manifested by Th1-type cytokine hyperactivity. In this study, the levels of Th1-type cytokines such as IL-2 and TNF-*α* were significantly higher than normal and Th2-type cytokines such as IL-10 were significantly lower than normal in both groups before treatment, indicating that the immune imbalance in CLT patients with hypothyroid may be dominated by Th1 cell immune response, which is consistent with the findings of the above study. After selenium supplementation, IL-2 and TNF-*α* levels decreased more significantly and IL-10 increased more significantly in the combined group, indicating that selenium can regulate the body's immune function, reduce the immune inflammatory response, and improve the condition of patients with CLT and hypothyroid. In previous studies, very little attention has been paid to the effects of selenium supplementation on the psychological and emotional aspects of patients during treatment. In this study, the SAS and SDS scales were used to assess patients' mood before and after treatment, and the results showed that both treatment regimens were able to improve patients' emotional state to some extent, but the combined treatment was superior to the single treatment, which may be related to the improvement of antithyroid antibody levels in patients. The results of this study also showed that the occurrence of adverse reactions in both groups was low and the difference was not significant, which further confirmed that LT4 combined with selenium supplementation treatment would not increase the occurrence of adverse events and the medication was safe.

In conclusion, this study found that selenium intervention therapy may help to reduce thyroid autoantibody titers, attenuate immune inflammatory responses, and improve mood in patients with CLT and hypothyroidism. The clinical outcome of patients treated with combined selenium supplementation was superior to that of the LT4 replacement therapy group alone, and selenium yeast may improve patient outcomes and halt disease progression with a high safety profile. However, this study still has shortcomings such as short observation time and not exploring the reasons for the poor efficacy of patients after selenium supplementation, which will be a problem for further research, as well as the efficiency and long-term efficacy of selenium in the treatment of CTL.

## Figures and Tables

**Figure 1:** Comparison of clinical efficacy between the control group and the combined group. Compared with the same index in the control group,  ^*∗*^*P* < 0.05.

**Figure 2:** Comparison of thyroid function between the control group and the combined group before and after treatment. (a) TT3 levels. (b) TT4 levels. (c) TSH levels. (d) TPOAb levels. (e) TGAb levels. Compared with the same group before treatment,  ^∧^*P* < 0.05; compared with the control group in the same period,  ^*∗*^*P* < 0.05.

**Figure 3:** Comparison of SAS and SDS scores between the control group and the combined group before and after treatment. (a) SAS scores. (b) SDS scores. Compared with the same group before treatment,  ^∧^*P* < 0.05; compared with the control group in the same period,  ^*∗*^*P* < 0.05.

**Figure 4:** Comparison of the levels of inflammatory factors between the control group and the combined group before and after treatment. (a) IL-2 levels. (b) IL-10 levels. (c) TNF*-α* levels. Compared with the same group before treatment,  ^∧^*P* < 0.05; compared with the control group in the same period,  ^*∗*^*P* < 0.05.

**Figure 5:** Comparison of the incidence of adverse reactions between the control group and the combined group.

**Table 1:** Comparison of basic information of patients in the two groups.

Information	Control group (*n* = 69)	Combined group (*n* = 69)	*z*/*t*/*χ*^2^ value	*P* value
Age (years, mean ± SD)	41.56 ± 6.13	42.63 ± 5.32	1.095	0.275
Disease duration (years, mean ± SD)	3.46 ± 1.70	3.52 ± 1.73	0.205	0.838
BMI (kg/m^2^, mean ± SD)	24.46 ± 3.15	24.09 ± 3.34	0.669	0.504
Gender (*n*, %)				
Male	21 (30.43)	23 (33.33)	0.134	0.715
Female	48 (69.57)	46 (66.67)		
Degree of goiter (*n*, %)				
Mild	17 (24.64)	19 (27.54)	−0.338	0.735
Moderate	38 (55.07)	37 (53.62)		
Severe	14 (20.29)	13 (18.84)		
Smoking history (*n*, %)	15 (21.74)	12 (17.39)	0.414	0.520
History of alcoholism (*n*, %)	20 (28.99)	18 (26.09)	0.145	0.703

## Data Availability

Data are available on request to the authors.
